The article "Health Promotion Combined with Psychological Care Improves Vestibular Function in Patients with Vestibular Neuritis" was published in 2022. Journal: Contrast Media Mol Imaging.

# Health Promotion Combined with Psychological Care Improves Vestibular Function in Patients with Vestibular Neuritis

**DOI:** 10.1155/2022/3780683

**Published:** 2022-08-13

**Authors:** Fan Peng, Rui Mei, Chanyuan Liu, Xiu Liu, Jing Xiong, Lu Lv, Fang Wang

**Affiliations:** ^1^Department of Rheumatology, Wuhan Traditional Chinese Medicine Hospital, Wuhan, China; ^2^Department of Acupuncture, Wuhan Traditional Chinese Medicine Hospital, Wuhan, China; ^3^Department of Medical Administration, Wuhan Mental Health Center, Wuhan, China; ^4^Department of Psychiatry, Wuhan Wuchang Hospital Nanhu District, Wuhan, China; ^5^Department of Obstetrics and Gynecology, Wuhan Wuchang Hospital, Wuhan, China; ^6^Department of Pharmacy, Wuhan First Hospital, Wuhan, China; ^7^General Affairs Section, Wuhan Mental Health Center, Wuhan, China; ^8^Psychosomatic Medical Ward, Wuhan Mental Health Center, Wuhan, China

## Abstract

This study aimed to explore the effect of health education combined with psychological care on patients with vestibular neuritis and the effect on their vestibular function. One hundred patients with vestibular neuritis admitted to our hospital from January 2019 to December 2020 were enrolled and divided into two groups by the random number: the control group (CG) (*n*= 53, health education) and the study group (SG) (*n*= 47, health education + psychological care). The Dizziness Handicap Inventory (DHI) scores, Berg Balance Scale (BBS) scores, depression scores (SDS), anxiety scores (SAS), satisfaction with care, compliance, incidence of falls, quality of life (QOF), and clinical symptom scores were compared between the two groups. Compared with the CG, the SG had a more significant reduction in DHI scores and SDS and SAS scores and a significant increase in BBS scores (*P* < 0.05). Compared with the CG, the SG had higher nursing satisfaction and compliance and a lower incidence of falls (*P* < 0.05). Nursing efficiency was higher in the SG than in the CG (*P* < 0.05). QOF scores were higher in the SG than in the CG (*P* < 0.05). Clinical symptom scores were lower in the SG than in the CG (*P* < 0.05). Health education combined with psychological care can improve vestibular function and bad mood, reduce the incidence of falls, improve the QOF, and result in high patient satisfaction and compliance, which should be widely promoted.

## 1. Introduction

Vestibular neuritis (VN) is a condition that causes vertigo, dizziness, dizziness, headache, visual sensitivity, nausea, and vomiting, affecting primarily a population of 20–60 years old [1]. The duration of acute vertigo in patients with VN often lasts for more than 1 day, and activation of herpes simplex virus potentially in the vestibular ganglion contributes to the development of VN [2]. Clinical data show that the incidence of VN is on the rise, with a prevalence of up to 9.0% of all vertigo manifesting disorders, adversely affecting the normal life and health of patients [3].

The article "Health Promotion Combined with Psychological Care Improves Vestibular Function in Patients with Vestibular Neuritis" was published in 2022. Journal: Contrast Media Mol Imaging.

Medication and rehabilitation are the main treatment options for VN, with significant short-term effects but poor efficacy in improving balance function [4]. In addition, some patients with vestibular vertigo experience anxiety and depression as well as other adverse emotions, which have an impact on the treatment effects [1]. Therefore, appropriate interventions should be explored clinically to improve negative emotions and promote recovery. Health education and psychological care are key to the clinical care of patients with VN and can be implemented according to changes in patients' cognitive abilities and psychological characteristics [5]. This study included 100 patients with VN admitted to our hospital from January 2019 to December 2020 to investigate the effects of health education and psychological care on vestibular function and clinical symptoms, aiming to improve patients' quality of life (QOF).

## 2. Materials and Methods

### 2.1. Baseline Data

One hundred patients with VN admitted to our hospital from January 2019 to December 2020 were enrolled. Inclusion criteria were (1) aged >18 years; (2) time from onset to admission <72 hours; (3) patients meeting the diagnostic criteria of VN; (4) patients with complete data and signed informed consent; (5) patients with normal cognitive function. Exclusion criteria were (1) patients with major organ injury; (2) patients unable to complete the follow-up; (3) patients with hearing impairment; (4) patients with severe diseases; (5) patients with neurological or central system impairment; (6) patients during pregnancy or lactation. The patients were randomly divided into two groups, i.e., the control group (CG) (*n*= 53) and the study group (SG) (*n*= 47). The baseline data of patients in the two groups were comparable (*P* > 0.05). Patients agreed to participate in the study and signed written informed consent before the study, and the study was approved by the Ethics Committee of Wuhan Mental Health Center. The study was conducted in accordance with the Declaration of Helsinki.

### 2.2. Nursing Methods

The CG was given health education. (1) Cognitive education: patients tend to have a low level of disease knowledge; nursing staff will explain the causes, clinical treatment, clinical manifestations, and the importance of care to the patients in easy-to-understand language. (2) Medication education: the patient was informed about the duration of medication, side effects, precautions, and expected therapeutic effects. Patients' drug allergy history before administration was inquired. (3) Rehabilitation catechism: moderate exercise is beneficial to recovery. Nursing staff provided advice on exercise intensity and duration via science education videos to improve patients' awareness and exercise compliance.

The article "Health Promotion Combined with Psychological Care Improves Vestibular Function in Patients with Vestibular Neuritis" was published in 2022. Journal: Contrast Media Mol Imaging.

In the SG, psychological care was provided in addition to health education. Patients received a warm welcome upon admission and were introduced about the hospital environment, which helped them accommodate the new environment more quickly and eliminate their negative emotions. Some patients kept eyes closed when receiving treatment, so communication should be carried out through gentle language. Patients' emotional changes should be observed and their needs should be listened to. Their subjective feelings should be cared about, and their questions should be answered patiently so that they can maintain a positive attitude towards life. Success stories should be shared to improve patients' self-confidence in treatment.

### 2.3. Outcome Measurement

DHI and BBS scores [6]: the vestibular function was evaluated by DHI and BBS. The DHI is a 25-item self-report questionnaire that quantifies the impact of dizziness on daily life by measuring self-perceived handicap. Item scores are summed. There is a maximum score of 100 (28 points for physical, 36 points for emotional, and 36 points for functional) and a minimum score of 0. The lower score indicated the lower severity of the balance disorder or vertigo. The BBS is a 14-item objective measure that assesses static balance and fall risk in adults, with each item consisting of a five-point ordinal scale ranging from 0 to 4, with 0 indicating the lowest level of function and 4 the highest level of function. The higher score indicated the better balance function.

SDS and SAS scores [7]: depression and anxiety were evaluated by SDS and SAS. Major depression or anxiety: >72 points, moderate depression or anxiety: 63–72 points, and mild depression or anxiety: 53–62 points. The lower score indicated the lower level of depression or anxiety.

Nursing satisfaction and adherence [8] were evaluated in terms of humanistic care, nursing attitude, health guidance, and nursing operation by our customized satisfaction questionnaire. Unsatisfied: satisfaction score <65, satisfied: satisfaction score ranged 65 to 80, and very satisfied: satisfaction score ≥80. Satisfaction was the ratio of the number of very satisfied and satisfied cases to the total number of cases, multiplied by 100%. Adherence covers 3 aspects: adherence to rehabilitation, adherence to nursing measures, and adherence to medication, with a total of 16 points. Poor adherence: 0–3 points, fair adherence: 4–9 points, and good adherence: 10–16 points.

The article "Health Promotion Combined with Psychological Care Improves Vestibular Function in Patients with Vestibular Neuritis" was published in 2022. Journal: Contrast Media Mol Imaging.

Effectiveness of care [9]: ineffective: no significant change in clinical signs and symptoms or further aggravation; effective: reduction of positional nystagmus or vertigo; significant improvement: disappearance of spontaneous nystagmus and nausea and vomiting and significant improvement of dizziness and headache. The effective rate was the ratio of the number of significant improvement and effective cases to the total number of cases, multiplied by 100%. The higher effective rate indicated the more ideal care effect.

QOF score [10]: the SF-36 scale was applied to evaluate patients' social, physical life, psychological, and somatic function, covering 0–100. The higher score indicated the better QOF.

Clinical symptoms score was evaluated in terms of balance disorder, vertigo, dizziness, headache, visual sensitivity, and nausea and vomiting. The lower score indicated the less severe symptoms.

### 2.4. Statistical Analysis

Statistical Package for the Social Sciences (SPSS) 19.0 (IBM, Armonk, NY, USA) was applied for data analysis. Count data were analyzed using the two-sided test. *P* < 0.05 was considered statistically significant. Quantitative data were expressed as (*x̅* ± *s*) and compared using the *t*-test, and ANOVA was used for comparison among three groups, followed by the LSD test. Qualitative data were tested using the *χ*^2^ test. Figures were produced using GraphpadPrism8.

## 3. Results

### 3.1. Comparison of DHI and BBS Scores

Before the intervention, there was no significant difference in DHI and BBS scores between the two groups (*P* > 0.05). After the intervention, the DHI scores decreased significantly, and the BBS scores increased significantly. Compared with the CG, the DHI scores were lower, and the BBS scores were higher in the SG (*P* < 0.05) (Table 1). It indicated that health education combined with psychological care improved patients' vestibular function.

### 3.2. Comparison of SDS and SAS Scores

Before the intervention, there was no significant difference in SDS and SAS scores between the two groups (*P* > 0.05). After the intervention, SDS and SAS scores decreased more significantly in the SG than in the CG (*P* < 0.05) (Table 2). It indicated that health education combined with psychological care relieved patients' adverse emotions.

### 3.3. Comparison of Nursing Satisfaction and Compliance

Nursing satisfaction and compliance were higher, and the incidence of falls was lower in the SG than in the CG (*P* < 0.05) (Table 3). It indicated that health education combined with psychological care improved nursing satisfaction and compliance.

The article "Health Promotion Combined with Psychological Care Improves Vestibular Function in Patients with Vestibular Neuritis" was published in 2022. Journal: Contrast Media Mol Imaging.

### 3.4. Comparison of the Nursing Effect

After the intervention, the nursing efficiency of the CG was 71.7%, and the nursing efficiency of the SG was 87.2%. The nursing efficiency of the SG was higher than that of the CG, showing statistically significant difference (*P* < 0.05) (Figure 1). It indicated that health education combined with psychological care resulted in high nursing efficiency.

### 3.5. Comparison of QOF Scores

Before the intervention, there was no significant difference in the QOF scores between the two groups (*P* > 0.05). After the intervention, the QOF scores in both groups increased significantly, but the increase in the QOF scores was more pronounced in the SG than the CG, and there was a difference in the QOF scores between the groups (*P* < 0.05) (Figure 2). It indicated that health education combined with psychological care improved the QOF.

### 3.6. Comparison of Clinical Symptom Scores

Before the intervention, there was no significant difference in the clinical symptom scores between the two groups (*P* > 0.05). After the intervention, the clinical symptom scores in both groups decreased significantly, and the clinical symptom scores in the SG decreased more significantly than those in the CG, showing statistically significant difference between the two groups (*P* < 0.05) (Figure 3). It indicated that health education combined with psychological care relieved the clinical symptom.

### 3.7. Comparison of DHI Scores

After the intervention, DHI-P, DHI-F, DHI-E, and DHI-total scores were significantly lower in the control and study groups, but the reduction in DHI scores was more pronounced in the SG than the CG (*P* < 0.05) (Figure 4). It indicated that health education combined with psychological care improved the severity of the balance disorder or vertigo.

## 4. Discussion

There is no definite study on the pathogenesis and causes of VN. Some scholars believe that the causative factors of VN are mainly autoimmune disorders and contemporaneous or preexisting bacterial and viral infections. VN is a nonspecific inflammatory disease that impairs vestibular function [11, 12]. Vestibular dysfunction involves both static and dynamic balance, with patients having static vestibular dysfunction experiencing spontaneous resolution of symptoms after 30 days of persistence [13]. Compared with static vestibular dysfunction, dynamic vestibular dysfunction can have a more serious impact on patients' QOF and prolonged the duration of symptoms. The pharmacological treatment can improve patients' body balance, vertigo, and vestibular dysfunction to a certain extent, but the treatment efficiency is low [14, 15]. In this study, health education combined with psychological care can relieve patients' adverse emotions.

The article "Health Promotion Combined with Psychological Care Improves Vestibular Function in Patients with Vestibular Neuritis" was published in 2022. Journal: Contrast Media Mol Imaging.

Patients with VN suffer from persistent vertigo and fear of exercise, leading to exacerbation of the disease and a vicious cycle that affects treatment outcomes [16]. This study, through cognitive, medication, and rehabilitation therapy, may improve patient motivation for rehabilitation and contribute to improved balance function and reduced severity of condition [17]. This study investigated the effect of the combination of health education and psychological care on the vestibular function of patients. The results showed that the SG had higher nursing efficiency, more significant reduction in DHI scores, and more significant increase in BBS scores than the CG (*P* < 0.05). It has been reported that compared with conventional nursing methods, nursing through the combination of health education and psychological nursing has a higher nursing efficiency, up to 92.5% [18], which is consistent with the results of this study. The results suggest that health education combined with psychological care can improve balance function and reduce the degree of vestibular dysfunction, which is a relatively feasible nursing method. Some VN patients with severe vertigo should be treated with sedative drugs, which can inhibit the process of vestibular compensation and increase the risk of mental illness [19]. Moreover, the duration of dynamic impairment of vestibular function is prolonged by maladaptive behaviors and secondary psychiatric disorders, increasing the difficulty of disease treatment and slowing recovery [20]. The above-mentioned factors tend to trigger adverse emotions. Through psychological intervention, the nurse actively communicates with the patient and gives verbal encouragement and affirmation so that the patient feels more care, improving their compliance [21, 22]. The study investigated the effect of health education combined with psychological care on patients' bad mood, and the results showed that the SDS and SAS scores were reduced more significantly in the SG than in the CG, and the nursing efficiency was higher in the SG than the CG (*P* < 0.05). The results showed that health education combined with psychological care could effectively relieve patients' anxiety and depression and increase patients' satisfaction with nursing, nursing attitude, health guidance, and nursing operation, and patients' rehabilitation process and medication compliance were significantly improved. Health education combined with psychological care can provide behavioral guidance and improve treatment compliance and adherence to medication, reducing the rate of accidental injury [23, 24]. The results of the present study showed that the QOF scores were much significantly higher, and clinical symptom scores were much significantly lower in the SG than the CG (*P* < 0.05). The results suggested that health education combined with psychological care plays a significant role in improving QOF and clinical symptoms.

The article "Health Promotion Combined with Psychological Care Improves Vestibular Function in Patients with Vestibular Neuritis" was published in 2022. Journal: Contrast Media Mol Imaging.

The study included eligible samples to explore the role of health education and psychological care on patients' vestibular function, dysphoria, nursing satisfaction, and compliance. Nonetheless, the study may have had an impact on the accuracy of the study due to the small sample size, the short study period, and the lack of an ongoing follow-up.

## 5. Conclusion

In conclusion, health education combined with psychological care for patients with VN is effective for improving vestibular function and dysphoria, reducing the incidence of falls and improving QOF, with high patient satisfaction and compliance, which should be widely promoted.

## Figures and Tables

**Figure 1:** Comparison of the nursing effect between the two groups, ^#^*P* < 0.05.

**Figure 2:** Comparison of quality of life scores, ^#^*P* < 0.05.

**Figure 3:** Comparison of clinical symptom scores, ^#^*P* < 0.05.

**Figure 4:** Comparison of DHI scores, ^#^*P* < 0.05.

**Table 1:** Comparison of DHI and BBS scores (*x̅* ± *s*).

Group	Number of cases	DHI score		BBS score	
		Preintervention	Postintervention	Preintervention	Postintervention
Control group	53	71.4 ± 5.4	31.1 ± 3.8	10.7 ± 2.1	31.1 ± 4.2
Study group	47	71.6 ± 5.3	23.8 ± 4.1	10.6 ± 2.3	40.9 ± 4.4
*t*	—	1.682	15.324	0.782	14.985
*P*	—	>0.05	<0.05	>0.05	<0.05

**Table 2:** Comparison of SDS and SAS scores (*x̅* ± *s*).

Group	Number of cases	SDS score		SAS score	
		Preintervention	Postintervention	Preintervention	Postintervention
Control group	53	58.4 ± 6.6	43.6 ± 5.8	64.1 ± 6.5	48.4 ± 3.8
Study group	47	57.7 ± 6.5	29.2 ± 2.1	63.8 ± 6.7	30.4 ± 3.5
*t*	—	0.524	16.354	1.087	18.175
*P*	—	>0.05	<0.05	>0.05	<0.05

**Table 3:** Comparison of nursing satisfaction, compliance, and incidence of falls (cases, %).

Group	Number of cases	Satisfaction	Adherence	Incidence of falls
Control group	37	31 (83.8)	29 (78.4)	7 (18.9)
Study group	41	39 (95.1)	38 (92.7)	1 (2.4)
*χ* ^2^	—	7.325	5.421	4.635
*P*	—	<0.05	<0.05	<0.05

## Data Availability

The datasets used and analyzed during the current study are available from the corresponding author on reasonable request.
